RETRACTED

# Effect of Sufentanil Combined with Nalmefene Assisted Surface Anesthesia on Transnasal Endotracheal Intubation Guided by Fiberoptic Bronchoscope

**DOI:** 10.1155/2022/5144875

**Published:** 2022-09-09

**Authors:** Zhanqi Zhao, Junting Zhang, Yuru Zhan, Zhongqun Wang

**Affiliations:** Department of Anesthesiology, The Third Affiliated Hospital of Qiqihar Medical College, Qiqihar, Heilongjiang 161000, China

## Abstract

In order to study the clinical effect of sufentanil combined with nalmefene in fiberoptic bronchoscopy tracheal intubation in airway patients, a method based on sufentanil combined with nalmefene-assisted topical anesthesia for fiberoptic bronchoscopy-guided nasotracheal intubation method is proposed. This method retrospectively analyzed 100 patients with difficult airways who underwent fiberoptic bronchoscope tracheal intubation in the Central Hospital from January 2021 to November 2021. The analysis results showed that compared with the control group, the patients in the study group had a significantly lower cough score, a higher Ramsay sedation score, a lower mean arterial pressure, and a lower number of patients with hypoxia (*P* < 0.05). There was no significant difference in postoperative hoarseness and sore throat between the two groups. Sufentanil combined with nalmefene has a better anesthesia effect and higher safety for bronchofiberscope intubation in patients with difficult airways.

## 1. Introduction

Fiberoptic bronchoscopic intubation is a common operation in clinical surgery, and it is often carried out in the awake state of patients. Anesthesiologists can inhibit the patient's stress response through sedation and anesthetic drugs, but for patients with a difficult airway, the application of anesthetic drugs needs to be carefully selected [1]. Research reports show that remifentanil, as an opioid analgesic, is the main anesthetic for fiberoptic bronchoscopy intubation. It has the characteristics of good analgesic effect, short action time, and good controllability. It has been widely used in anesthesia induction and intraoperative maintenance. Sufentanil is a receptor agonist recently used in clinics [2]. It has sedative and analgesic effects (Figure 1) and has no inhibitory effect on respiration. It can significantly reduce the amount of anesthetic required to induce and maintain anesthesia, promote the stability of catecholamine hemodynamics, and effectively reduce the stress related to anesthesia and surgery [3]. Especially for patients with difficult respiratory tract, when intubation with a fiberoptic bronchoscope, patients have a large stress response and uncontrollable. Therefore, Sufentanil is a better choice of narcotic drugs. This study observed the clinical effect of Sufentanil combined with remifentanil in awake endotracheal intubation. It is reported as follows:

RETRACTED

## 2. Literature Review

Fiberoptic bronchoscopy is the most commonly used invasive and invasive examination in clinical diagnosis and treatment of lung diseases [4]. Mechanical stimulation during the examination will cause airway spasms and reflex contraction, and induce patients to have a repeated cough, suffocation, laryngeal spasm, and so on. It leads to a decrease in blood oxygen saturation, an increase in heart rate and even serious arrhythmia, and an increase in blood pressure, which not only increases the operation difficulty of endoscopists but also increases the risk of bronchial mucosal injury and cardiovascular and cerebrovascular accidents [5]. In this examination, the problems to be faced by anesthesia management include (1) Most of the patients are the elderly with chronic lung disease, poor lung reserve function, and low tolerance to hypoxia, often combined with multisystem diseases and high anesthesia risk. Adequate preoperative preparation, control of blood pressure and blood glucose, and monitoring of blood oxygen saturation are needed to reduce the risk of adverse events. (2) Some patients will suffer from hypoxemia due to lung diseases, and also cannot tolerate severe hypoxia [6]. How to ensure the oxygen in the operation process of these patients is a problem that we need to pay attention to. (3) During the examination, anesthesiologists and endoscopists share the airway, which increases the difficulty of airway management.

Propofol and opioids are commonly used in clinical anesthesia for bronchoscopy. Propofol is the most commonly used intravenous anesthetic in the clinic [7]. It has the advantages of fast onset, strong controllability, stable hemodynamics, and rapid postoperative recovery. It is widely used in painless treatment. At the same time, because of its poor analgesic effect and obvious inhibitory effect on the cardiovascular system, propofol and opioids are often used in the clinic to make up for the lack of analgesic effect and reduce the side effects of a single drug. Both drugs can inhibit respiration and circulation [8]. The combination of the two drugs will aggravate respiratory inhibition and severe fluctuation of hemodynamics, and significantly increase the risk of airway management. Sen et al. and others showed that fentanyl caused nausea and vomiting by stimulating the chemical sensing area of the fourth ventricle; respiratory depression due to reduced central stimulation caused by elevated carbon dioxide; it also causes rigidity of thoracic muscles, choking and coughing in patients, which can induce airway spasm and asthma attack; and the recovery of postoperative orientation is poor and easy to be restless [9]. Ezg et al. and others through the research on the application of sufentanil and propofol combined anesthesia in outpatient surgery of elderly patients, believe that they have superposition and synergy, which can deepen the anesthetic effect, but the incidence of adverse reactions increases and is dose-dependent [10].

RETRACTED

## 3. Experimental Analysis

### 3.1. Subjects

A retrospective analysis of 100 patients with airway difficulties who underwent fiberoptic bronchoscope tracheal intubation in the central hospital from January 2021 to November 2021. They were divided into observation groups and control groups, with 50 patients in each group. The patients were classified as grades I1∼II by the American Society of anesthesiologists and grades I–IV by Malampatti. There were 21 males and 29 females in the observation group, aged 34–63 (40.3 ± 14.5) years and weighing (66.5 ± 18.5) kg; there were 18 cases of mandibular fracture, 10 cases of laryngeal cancer, 9 cases of temporomandibular joint fusion, 9 cases of small jaw deformity and 4 cases of tongue hemangioma. In the control group, there were 24 males and 26 females, aged 35–61 (38.9 + 12.4) years and weighing (65.1 + 14.9) kg; there were 19 cases of mandibular fracture, 11 cases of laryngeal cancer, 10 cases of temporomandibular joint fusion, 8 cases of small jaw deformity and 2 cases of tongue hemangioma [11]. Exclusion criteria were as follows: Patients with severe hypertension, arrhythmia, asthma, nervous system diseases, and long-term history of sedative and analgesic drugs before operation; family genetic history; patients with severe liver and kidney dysfunction; and those with a history of drug allergy. There was no significant difference in general clinical data such as gender, age, and weight between the two groups (*P* > 0.05).

### 3.2. Experimental Method

The patient fasted 6 hours and drank 4 hours before the operation. After entering the room, in the supine position, establish peripheral venous access, monitor the patient's heart rate, blood oxygen saturation, systolic blood pressure, and diastolic blood pressure, and give nasal catheter oxygen inhalation of 3 L/min [12].

#### 3.2.1. Anesthesia Method

The two groups of patients were respectively given oxycodone hydrochloride injection 0.1 mg/kg + nalmefene 0.5-0.6 *μ*g/kg (oxycodone hydrochloride group) and sufentanil injection 0.06–0.1 *μ*g/kg + nalmefene 0.5-0.6 *μ*g/kg (sufentanil group). The infusion of nalmefene was completed within 10 minutes, and both groups underwent cricothyroid membrane puncture and intratracheal anesthesia with 1.5 ml of 1% tetracaine solution. About 5 minutes later, a bronchoscopy was performed. All the surgeons used transnasal operation, and before the operation, 1 ml of 2% lidocaine was instilled into the nasal cavity for mucosal surface anesthesia, and 3 ml of 2% lidocaine was injected into the glottis and the left and right bronchi respectively for local anesthesia [13].

RETRACTED

#### 3.2.2. Alert/Sedation Scoring Standard and Anesthetic Effect Grading Standard

Alert/sedation (OAA/s) scoring standard: 5 points refer to the rapid response to the call of normal tone; 4 points refer to cold response; 3 points refer to the response to loud and repeated name calls; 2 points refer to a reaction to slight shaking of body parts; 1 point refers to no response to shaking the body; and a score of 0 means that there is still no response to relatively hard things such as pinching the earlobe. The grading standard of anesthetic effect 9 patients. Excellent: the glottis is well opened, the entry into the mirror is smooth, the patient is quiet, the cooperation is good, there is no nausea and cough, and the examination is smooth [14]; it may be that the glottis is not opened well, the entry into the mirror is not smooth enough, there is nausea reaction, the cough is serious during operation, and lidocaine needs to be supplemented for many times to strengthen the effect of local anesthesia; it means that the glottis is not easy to open, the access to the mirror is not smooth, the patient is disgusting, accompanied by severe choking and suffocation, and the examination cannot be completed. Satisfaction survey: the whole process is satisfied if there is no obvious discomfort; although there is discomfort, tolerable is basic satisfaction; what is unbearable is dissatisfaction. Investigation of willingness to accept the second examination: ask the patient how he feels during the examination and whether he is willing to accept the second examination under this anesthesia if necessary.

#### 3.2.3. Intraoperative Treatment

If the heart rate is lower than 50 beats/min during the operation, give an intravenous injection of atropine injection 0.25 mg; if the decrease of systolic blood pressure exceeds 30% of T0, intravenous injection of m-hydroxylamine 0.5 mg; when both appeared at the same time, dopamine 3 mg was injected intravenously; if the patient has breath holding, body movement or severe choking cough during operation, resulting in tachycardia (> 120 beats/min), high blood pressure (SBP > 160 mmHg or DSP > 100 mmHg) and SpO_2_ < 90%, the bronchoscope can retreat to the main airway, and the patient can be instructed to breathe deeply and increase the oxygen flow appropriately [15]. At the same time, the operator can give 2 ml of 2% lidocaine local spray anesthesia, and reduce heart rate and blood pressure if necessary. After the anesthesia takes effect and the patient's vital signs are stable, continue the examination and operation.

RETRACTED

#### 3.2.4. Observation Indicators

Record the examination time of the two groups of patients; HR, SpO2, SBP, and DBP were recorded at 6-time points under quiet state (T0), before entering the lens (T1), immediately after glottis (T2), 5 min (T3), 10 min (T4) after glottis, and two minutes (T5) after going out of the lens; observe and record the adverse reactions during the examination, such as breath holding, body movement, hypotension, severe choking, as well as nausea and vomiting within 24 hours after operation; the patients were assessed with alert/sedation (OAA/S) score and anesthetic effect grade, and followed up on satisfaction and willingness to accept re-examination if necessary [16].

### 3.3. Statistical Analysis

Spss19.0 statistical software was used to analyze all the result data. [17] The measurement data were expressed by mean ± standard deviation (*x* ± *s*). The comparison between the two groups was performed by *t*-test, and the comparison within the group was performed by one-way ANOVA; chi-square test was used to compare the counting data. The difference was statistically significant (*P* < 0.05).

### 3.4. Result Analysis

All patients in this study did not withdraw from the trial for any reason and successfully completed awake endotracheal intubation after trying to intubate 1-2 times. There was no significant difference in the general data [18] between the two groups, as shown in Table 1.

The mean arterial pressure, heart rate, and Ramsay sedation score were compared between the two groups at each time point. During anesthesia, no patient had severe hypotension (MAP < 60 mmHg, 1 mmHg = 0.133 kPa) or bradycardia (HR < 50 beats/min), see Figures 2 and 3. The MAP and HR at T2. T in the control group were higher than those at T. The MAP and HR at T. T2 and T3 time points in the sulmeifen group were higher than those in T. decreased (*P* < 0.05). Dexmedetomidine group T, T2. T: Ramsay sedation score at time point compared with T. time increased (*P* < 0.05), but there was no significant difference between all-time points in the control group. Compared with the control group, the MAP at T2 and T3 in the sumeifene group decreased (*P* ≤ 0.01), while the HR at T1, T2, and T3 in the sumeifene group decreased (*P* ≤ 0.01), and the Ramsay score increased (*P* < 0.05).

There was no significant difference in respiratory monitoring indexes and endotracheal intubation between the two groups (Table 2).

RETRACTED

In a comparison of postoperative complications between the two groups, there was no significant difference in the number of cases of hoarseness and throat pain between the two groups (Table 3).

## 4. Discussion

Fiberoptic bronchoscope (FBS) assisted transnasal endotracheal intubation is a safe and effective method to establish an artificial airway. However, it is easy to induce a strong stress response, and then cause the activation of the sympathetic adrenocortical system, resulting in the increase of catecholamine levels in the blood, which can lead to strong changes in hemodynamics; at the same time, it may also leave a bad memory for patients, and even lead to serious complications [19]. Therefore, it is of great significance to find a safe and effective method of sedation and analgesia. Sufentanil is a new type of highly selective *a*_2_ adrenergic receptor agonist. It acts on *a*_2_ adrenergic receptors in the brain and spinal cord inhibits neuronal discharge and produces sedative, analgesic, and sympathetic effects. In addition, some scholars have safely applied Sufentanil to FBS-guided difficult endotracheal intubation under conscious sedation and achieved a good conscious sedation effect [20].

The difficult airway is always a big challenge for anesthesiologists in the process of anesthesia, especially the unexpected difficult airway before anesthesia. In most cases, it is reasonable to complete intubation in patients' sleep after anesthesia induction. But in some patients, conscious intubation is the safest [21]. Domestic hospitals routinely implement awake endotracheal intubation to minimize the risk of “unable to ventilate and intubate.” However, endotracheal intubation in an awake state is a strong stressor for patients, both physically and psychologically. Therefore, conscious intubation requires good sedation and analgesia, does not inhibit breathing, and reduces stress reactions such as choking and severe fluctuation of circulation during intubation and postoperative psychological trauma as much as possible. Sufentanil is a highly selective *α*^2^ receptor agonist, which plays a sedative role by reducing the release of inhibitory nerve cells from locus coeruleus to the ventral lateral preoptic nucleus, resulting in increased release of *γ*-aminobutyric acid (GABA); it also produces spinal cord level analgesia through the descending inhibitory pathway originating from the midbrain [22]. Because Sufentanil has a strong sedative effect and does not affect respiration, it is often used for sedation on various occasions, especially in patients in the intensive care unit (ICU). The initial purpose of this study is to observe the application of Sufentanil in awake intubation based on its characteristics.

RETRACTED

In this study, the mean arterial pressure and heart rate in the study group were significantly lower than those in the control group (*P* < 0.05). Map and HR in the control group were higher than those before anesthesia, while map and HR in the Sufentanil group were significantly lower than those before anesthesia. This shows that Sufentanil can well inhibit the strong stress response of endotracheal intubation, which is significantly better than fentanyl. It is more suitable for conscious endotracheal intubation in elderly patients with more cardiovascular diseases [23]. At the same time, it is worth noting that after the application of Sufentanil, it is necessary to closely monitor the changes in hemodynamics to prevent excessive reduction of blood pressure and heart rate, resulting in unnecessary cardiovascular accidents in elderly patients. When anesthesiologists choose sedative and analgesic drugs for conscious endotracheal intubation, whether respiratory depression will occur is still one of the key considerations. In this study, there was no significant difference in respiratory rate between the two groups. After a 24-hour follow-up, there was no significant difference in hoarseness and throat pain between the two groups [24]. Although the number of patients with hypoxia in the Sufentanil group was significantly less than that in the control group, SpO_2_ < 90% was still found in 3 patients. This suggests that the clinical application of Sufentanil for conscious sedation still needs to be closely monitored for respiratory function.

It is reported that the peripheral or intravenous application of Sufentanil can increase the Ramsay sedation score and reduce the bispectral index of EEG in patients under regional block anesthesia and intraspinal anesthesia. The results also showed that the Ramsay Sedation score in the Sufentanil group was significantly higher than that in the control group; the choking reaction of patients in the Sufentanil group during intubation was significantly better than that in the control group, indicating that Sufentanil can not only provide sufficient sedation for elderly patients but also inhibit the harmful stimulation of intubation operation to tracheal mucosa [25]. However, different from some studies at home and abroad, there is no significant difference between the two groups in the degree of tolerance to the endotracheal tube after intubation, and most elderly patients have good tolerance to endotracheal tubes. This may be related to the use of detailed preoperative communication, good tracheal mucosa and throat surface anesthesia in this study, or the large dose of Sufentanil in this study protocol. 1-151 to sum up, Sufentanil can effectively inhibit the violent fluctuation of circulation and provide good sedation when used for conscious endotracheal intubation in elderly patients, which is worthy of reference and application by clinicians.

RETRACTED

## 5. Conclusion

Propofol and etomidate are widely used in outpatient anesthesia, mainly for multi-disciplinary indoor endoscopy and outpatient short surgery, so as to achieve antianxiety, sedation, reduce patient discomfort, reduce stress response caused by stretch reflex, etc. Propofol has a high inhibitory effect on the circulatory system. On the one hand, it can dilate peripheral blood vessels, on the other hand, it has a direct effect on the myocardium, which can cause obvious hypotension and a large cardiac load. At the same time, propofol inhibited the respiratory system to a certain extent, resulting in the decline of tidal volume and respiratory rate. The elderly and weak patients are prone to apnea after medication, which requires anesthesiologists to pay attention to the changes in blood oxygen saturation. In recent years, many studies at home and abroad have confirmed that the hemodynamic stability and respiratory stability after etomidate anesthesia in painless endoscopy are better than propofol. However, etomidate usually causes myoclonus, which may disturb the endoscopic operation, and the incidence of nausea and vomiting is higher after the examination. Sufentanil can not only reduce the incidence of myoclonus but also significantly inhibit the occurrence of nausea and vomiting. While reaching and maintaining a sufficient level of sedation, the unique drug characteristics of Sufentanil make its sedative affect a physiological sleep mode that is easy to be awakened by auditory stimulation. This mechanism plays its special sleep role through the internal sleep induction and maintenance mode, which has a slight impact on respiration, increases the satisfaction of outpatient examination, and ensures the safety of outpatient endoscopic operation during the perioperative anesthesia period.

## Figures and Tables

**Figure 1:** Drug labor.

**Figure 2:** Comparison of mean arterial pressure sedation scores between the two groups at each time point.

**Figure 3:** Comparison of heart rate scores between the two groups at each time point.

**Table 1:** Comparison of general data between the two groups.

Group	Age (years)	Height (L/em)	Number of gears (kg/m^2^)	Gender (male/female)
Oxycodone hydrochloride group	65 ± 6.4	167 ± 9.1	24.1 ± 4.0	51/69
Sufentanil group	67 ± 8.1	164 ± 7.2	26.2 ± 6.3	49/61
Statistical value	0.52	1.50	0.89	0.07
*P* value	0.304	0.312	0.756	0.800

RETRACTED

**Table 2:** Comparison of respiratory monitoring indexes and endotracheal intubation between the two groups.

Group	Respiratory rate	Number of hypoxic cases	Degree of choking and number of cases	Degree of choking and number of cases
Oxycodone hydrochloride group	11 ± 3.4	51	(1/2/3/4)	(1/2/3/4)
Sufentanil group	10 ± 3.9	15	17/10/3/0	17/10/3/0
Statistical value	0.68	5.81	25/5/0/0	25/5/0/0
*P* value	0.545	0.038	3.34	3.34

**Table 3:** Comparison of postoperative complications between the two groups.

Group	Hoarseness	Sore throat
Control group	30	40
Oxycodone hydrochloride group	23	35
Sufentanil group	0.213	0.092
*P* value	0.740	0.765

## Data Availability

The data used to support the findings of this study are available from the corresponding author upon request.
